# Monitoring the Emotional Response to the COVID-19 Pandemic Using Sentiment Analysis: A Case Study in Mexico

**DOI:** 10.1155/2022/4914665

**Published:** 2022-05-18

**Authors:** Edgar León-Sandoval, Mahdi Zareei, Liliana Ibeth Barbosa-Santillán, Luis Eduardo Falcón Morales, Antonio Pareja Lora, Gilberto Ochoa Ruiz

**Affiliations:** ^1^School of Engineering and Sciences, Monterrey Institute of Technology and Higher Education, Monterrey, Mexico; ^2^Universidad de Alcalá, Alcalá, Spain

## Abstract

The world is facing the COVID-19 pandemic, leading to an unprecedented change in the lifestyle routines of millions. Beyond the general physical health, financial, and social repercussions of the pandemic, the adopted mitigation measures also present significant challenges in the population's mental health and health programs. It is complex for public organizations to measure the population's mental health in order to incorporate it into their own decision-making process. Traditional survey methods are time-consuming, expensive, and fail to provide the continuous information needed to respond to the rapidly evolving effects of governmental policies on the population's mental health. A significant portion of the population has turned to social media to express the details of their daily life, rendering this public data a rich field for understanding emotional and mental well-being. This study aims to track and measure the sentiment changes of the Mexican population in response to the COVID-19 pandemic. To this end, we analyzed 760,064,879 public domain tweets collected from a public access repository to examine the collective shifts in the general mood about the pandemic evolution, news cycles, and governmental policies using open sentiment analysis tools. Sentiment analysis polarity scores, which oscillate around -0.15, show a weekly seasonality according to Twitter's usage and a consistently negative outlook from the population. It also remarks on the increased controversy after the governmental decision to terminate the lockdown and the celebrated holidays, which encouraged the people to incur social gatherings. These findings expose the adverse emotional effects of the ongoing pandemic while showing an increase in social media usage rates of 2.38 times, which users employ as a coping mechanism to mitigate the feelings of isolation related to long-term social distancing. The findings have important implications in the mental health infrastructure for ongoing mitigation efforts and feedback on the perception of policies and other measures. The overall trend of the sentiment polarity is 0.0001110643.

## 1. Introduction

As the world faces new challenges with the COVID-19 (Coronavirus Disease 2019) pandemic, it becomes increasingly crucial for governments, public, and private organizations to consider the public's well-being in the decision-making process. The COVID-19 pandemic strongly impacts the population's physical health, a decisive factor in the current decision-making process. However, the COVID-19 pandemic also presents challenges in the emotional and psychological well-being of individuals.

This raises the need to collect physical health-related data and build dashboards showing critical information, making it easily accessible. Equally important is the need to get day-to-day data on the pandemic progression regarding ongoing infection rates and fatality, among other statistics. However, another important dimension, which we refer to as emotional health, has not been properly studied in Mexico, and no instruments for measuring it have been developed, which has long-term implications for the population's general well-being. These reasons highlight the need for a large-scale, resilient system to perform sentiment analysis in large, continuous datasets, such as Twitter traffic.

Sentiment analysis refers to a group of natural language processing techniques that allow extracting affective indicators from raw text to determine the polarity of a given tweet, that is, if the tweet expresses a positive or negative emotion. To measure the sentiment polarity of tweets, we employ VADER (Valence Aware Dictionary and sEntiment Reasoner) [1]. VADER is an open-source, rule-based tool that is able to recognize common terms, idioms, jargon, and more complex grammar structures such as punctuation, negations, and abbreviations that are commonly employed in social media platforms. VADER uses a curated lexicon of over 7,500 common terms rated by ten independent humans. VADER has been extensively validated for Twitter-based content, showing good results in terms of accuracy for tweets in several sentiment analysis tools [2]. For the reasons mentioned, we have selected this analyzer for this study.

Acquiring and processing this amount of information is not an easy task, for this is a perfect example of the challenges encountered by the three Vs. of Big-Data: Volume, Variety, and Velocity [3]. Here, we adhere to the most common definition of big data based on “the three Vs,” used in [3] and first introduced by [4]. But there are multiple definitions containing different aspects of these architectures, such as analysis, value, computer power, visualization, variability, and veracity, among various others. An in-depth description of these definitions is described by [5], but suffice to say that this research work adheres to the big data by most definitions.

This presents several problems, such as those listed as follows:

- Acquiring feedback on the emotional state is both expensive and time-consuming.
- Having that data available presents a significant challenge in processing capabilities and time to get feedback.
- Building such systems is costly, regardless of volume variations that may occur in the data.

Traditional survey methods for gathering information are prohibitive; besides the high expense, they require a significant amount of time to gather feedback on a small portion of the population, providing information on discrete periods rather than a continuous flow. Twitter is a mature, well-established, and popular microblogging service that offers users a platform to share their opinions, conversations, reviews, and other information. A large corpus for heterogeneous data was collected by [6], which we will refer to as the COVID-19 Twitter chatter dataset. It includes raw text, tweet metadata, images, videos, URLs, and popularity. This corpus is an excellent candidate for performing sentiment analysis to follow public opinion on any given topic or event but presents several challenges, including high computing resources needed for the research and a curated, well-defined training corpus. Furthermore, the advances in technology nowadays allow the processing of data in large volumes, at a fast velocity, and from numerous heterogeneous sources, making possible the analysis of sentiments on a near real-time basis [7].

Several studies have used sentiment analysis on Twitter in financial, political, and social, among other applications [8]. Sentiment analysis research makes extensive use of Twitter-related traffic, partly due to the high volume [9], high availability, and the limit of 280 characters per entry [10]. A survey shows that it is feasible to build such systems running on private clouds relying on the Hadoop tech stack. However, these systems are expensive: they require a significant up-front investment, require effort to set up and maintain, and fail to scale according to the demand [3]. Lastly, the validity of using these techniques to measure the subjects' emotional well-being has been under study by [11, 12].

Our study analyzes the sentiment polarity of tweets related to the COVID-19 pandemic posted by users in Mexico to assess the emotional well-being of the population and its evolution during the year 2020. Next, we present a survey of similar or related systems, highlighting for each one of them the technology used, their advantages, and their shortcomings, hoping to build upon them rather than creating a prototype from scratch.  Table 1 displays a summary of these systems, showcasing that most prototypes are supported by Apache Hadoop technologies for streaming and batch data processing. While these present good results, they also lack flexibility and scalability, resulting in high maintenance costs. We reviewed a collection of similar studies, summarized in Table 2, where we found them to utilize a small dataset, either in volume or in the length of the analyzed time frame. In general, only tweets written in English were accepted, restricted to the US, with just a couple of exceptions. For example, in [20], the studied tweets were restricted to those that originated in Australia only, in contrast to the survey made by [23], which uses a global dataset. Each study implements its own filtering criteria, making comparing results difficult, especially since they have not made their data sets public. We found key differences in the methodology as well. This study is most aligned with [23], which performs time series analysis over the dataset. The rest uses panel data analysis, separating the pandemic, in a fixed set of stages, either predefined or found through clustering using LDA (Latent Dirichlet Allocation) for topic discovery. Regardless of the details, an emerging pattern is to discover popular topics, report an average sentiment polarity over the cluster of tweets for the given subjects, or find the most influential users and focus the analysis on the timelines of such users. Instead of following this pattern, for this study, we diverge in the following points:

- Our study spans the study for a year-long worth of data, forcing us to deal with an extensive dataset.
- We make use of an already defined, publicly available dataset.
- This work focuses on the geographical area of study in Mexico, including tweets in both English and Spanish.
- We employ time series analysis in general to better measure the evolution of the public perception of the pandemic.
- We remove all confidential, sensitive, and personally identifiable information from the metadata available, making it impossible to analyze a particular individual's timeline.

It is worth noticing that important dates have a strong impact on the population's emotions. We focused the analysis on only those events where official announcements were made available nationwide. The information about these events was taken directly from [27, 28] and the official reports from the public health department, such as [29]. Details on these events are elaborated in the experiments section.

The outline of this work is as follows. This introduction section included a brief background of the problem and a literature review of similar applications and studies. The following section, Method, describes the followed methodology of the research, covering the data acquisition and general flow of the analysis, details of the time series models constructed and relevant events in different periods and experiments executed, and the technical elements of the architecture implemented to achieve this goal. Next, the results are presented along with relevant findings and figures. Finally, we conclude with a discussion, describing the observed phenomena and drawing the conclusion from the data and highlighting the strong points, limitations, and next steps of this work.

## 2. Method of the Emotional Response to the COVID-19 Pandemic Using Sentiment Analysis: A Case Study in Mexico

This section describes the data gathering process, the data processing performed, the technical solution's general architecture, and the analysis performed on the data gathered.

### 2.1. Data

We used a large dataset of tweets collected from an open-access repository of global COVID-19 related tweets, designed to collect every tweet posted that is somehow related to the pandemic in a diverse variety of geographic locations. It includes timeline metadata, allowing us to perform social network analysis on this *COVID-19 Twitter chatter dataset*. This repository provides a list of Tweet IDs, its geographical location, and detected language, utilizing the following schema: *[tweet_id, date, time, lang, country_code]*. However, we encountered schema inconsistencies over time. For example, the annotation of *country_code*, which is necessary for filtering before requesting a tweet lookup, was not introduced until the second half of the year, and even so, a vast number of tweets lack this metadata annotation.

For this reason, we had to load them via Twitter's public API in order to filter out tweets originated from outside Mexico, which may leave data out from those users who choose not to share their location. We used this information to download each tweet in Mexico, discarding all other metadata provided by Twitter's API for privacy reasons. Specifically, we retrieved COVID-19-related tweets posted in Mexico from February 1, 2020, through December 31, 2020. All tweets were scrubbed of any personally identifiable information to ensure user's privacy and comply with ethical, social media use practices, resulting in the following simplified schema: *full_text, id*. It is worth mentioning that this dataset includes tweets in both English and Spanish, for a large part of the population engages in social media in English.

Figure 1 shows the data ingestion pipeline, for which we used the regular lookup API (https://api.twitter.com/2/tweets?ids=[…]). However, this design allows for this API to be swapped for other endpoints, such as the search endpoint, allowing data consumption as a near real-time data stream without the need to perform any further changes to the existing solution. Note that the resulting sample size for the dataset exceeds the mean utilized by a recent scoping survey [30] on social media analytics for public health by several orders of magnitude (*n*=20,000 compared to ours, *n*=2,142,800), resulting in an ample sample into which to conduct this analysis. Previous studies, summarized in Table 2, used large-scale sentiment analysis to accurately predict the public's mood and how it applies to several domains, including those of emotional and psychological well-being [11]. Following the sentiment polarity determination, we pass the data through several analyses explained in detail in the section *Sentiment Analysis of the Emotional Response to the COVID-19 Pandemic in Mexico* and *Procedure*, performed in weekly averages, rolling 3-day averages, and daily smoothed averages. This last technique was found to describe best the trends found in the time series.

### 2.2. General Architecture Implemented in Google Cloud Platform (GCP)

This work has several technical requirements that need to be fulfilled in order to succeed. First, the system needs to ingest large amounts of data in the smallest possible quantity of time while having the flexibility to change the parameters of the data consumed and cutting costs by adjusting the scale needed according to the volume of data.

Secondly, the system also needs to maintain user's privacy and keep the data secure at all times. And finally, it is also desirable to use a modern technology stack such that we can exploit state-of-the-art deep-learning-based language models and implementation with low-level optimization for the data processing. These requirements are satisfied by implementing cloud technologies, a serverless architecture, and industry-standard ML-ops practices.

Thus, the system was implemented on top of Google Cloud Services (GCP) for its dynamic scaling of managed infrastructure and tight integration with the *TensorFlow* technology stack, enabling dynamic scaling, loose coupling, and managed microservices.  Figure 2 shows the general architecture of the solution, which can be seen it is separated into several modules. The general data flow is as follows:

- Data are ingested directly from Twitter, using the identifiers provided by the *COVID-19 Twitter chatter dataset* and the public query API provided by Twitter.
- The queried tweet is posted in Pub/Sub, where it is written directly in cloud storage for possible future reference and debugging.
- Pub/Sub feeds this data entry into a microservice, which evaluates the tweet polarity using a VADER [1] implementation written in *Python*, and posts the results again in Pub/Sub to be fed into BigTable for final consumption. A brief VADER description can be found in Subsection 2.3.
- The data are now ready for consumption by a managed Dataproc instance with two different approaches:
- Periodic batch jobs, which collect daily aggregations. These aggregations are also stored in cloud storage for easy access.
- Jupyter notebooks for manual data exploration.
- A third hook can be placed here for generating near real-time visualizations of the gathered data. We used the daily aggregations generated by the batch jobs for this study.

All the code was implemented using standard *Python* 3.6 and its data-focused libraries. The language models used for polarity calculation were implemented in TensorFlow. TensorFlow enables consuming state-of-the-art language models as a service, decoupling this architecture from the rest of the solution and allowing the implementation of an automated ML-ops flow to inject updates and model changes. Note the clear separation of operations performed to the ingested data and that this flow allows for ingesting data as streams, thus allowing using this solution as a decision-making tool by providing near real-time data processing. The operations performed on the data can be described in three steps: preprocessing, sentiment polarity calculation, and general aggregation. The preprocessing performed is data cleanup, for the language model itself handles any operations required by the language models, such as tokenization. The cleanup performed follows the standard practices and as such, they are not enumerated in this work.

### 2.3. Sentiment Analysis of the Emotional Response to the COVID-19 Pandemic in Mexico

To measure the sentiment polarity of tweets, we employ VADER. This open-source, rule-based tool is robust enough to be able to handle commonly employed complex grammar structures in social media platforms. It is important to note that the word virus, and its variations, is not included in the training lexicon; thus, this particular term has no impact on the sentiment polarity evaluation. The sentiment taxonomy employed by VADER covers two dimensions, ranging from positive to negative and from objective to subjective. However, this score is represented as a single numerical value, going from −1 to 1, where 1 is very positive, −1 is very negative, and 0 is neutral or completely objective. We can find a summary of these other solutions, applied in somewhat similar circumstances, in Table 2.

### 2.4. Procedure

Data are directly consumed using the Twitter public API, which is then put into hard storage as a simple comma-separated (.csv) file. This action automatically triggers change events that then feeds the entries into a data pipeline, making this easy to swap them for tweet feeds. This also helped us mitigate Twitter's API limitations by consuming them using multiple clients and feeding the results into a single location. Data then are cleaned and stored into a large non-sql database, in our case, into BigTable. From BigTable, we query data for exploration, experimentation, or model training, but we use data triggers to feed them into the sentiment polarity calculator, ending in another BigTable instance. This final instance is used as a source for aggregation and analysis, generating daily aggregates. This data pipeline produces the processing, cleaning, and experimentation needed, giving access points in each processing stage for experimentation or visualization.

Sentiment can change over time as individuals discuss different topics or because of changes in the emotional state of the individuals. To mitigate the impact of the former in the study, we utilized a COVID-19 curated dataset, the *COVID-19 Twitter chatter dataset*, which focuses on topics related to the pandemic. We then used daily sentiment scores for the Twitter corpus ranging from February 1 to December 31, 2020. We determine change-points in the time series of the daily average VADER sentiment polarity to identify significant sentiment changes during this time period. For the time series analysis, we followed the standard methodology. We start by denoising the series, for which we opted for a moving average of seven days as we also found a strong weekly seasonality in the data.

Next, data are detrended by fitting a regular time series model, for which several partial autocorrelation tests were performed to find a good initial parameter approximation and validate the model. Residuals and box testing reveal a good fit of the model, resulting in a *p* − value < 2.2*∗*10^−16^. These steps were repeated for several aggregation statistics, keeping relevant both the mean and the standard deviation as they summarize well the behavior observed in the data. The next section covers more details on the experiments and the results obtained from this analysis.

## 3. Experiments

We performed sentiment analysis on COVID-19 related tweets posted in Mexico from February 1, 2020, to December 31, 2020, forming a corpus of 760,064,879 tweets, which after preprocessing and filtering came to a total of *n*=2,142,890 utilized tweets, retrieved from the *COVID-19 Twitter chatter dataset*.

Table 3 shows monthly summary of the sentiment polarity for a given month. Please note that the ranges of values go from −1 (i.e., very negative) to 1 (i.e., very positive), where 0 is considered a neutral value or a completely objective tweet.

However, the time series analysis we performed on the data was with a daily granularity. From there, a box-test showed a *p* − value < 2.2*e* − 16, indicating a high probability of encountering auto-correlations in the data. This led to further exploration using partial ACF (Autocorrelation Function), summarized in Table 4. Here, we observe strong indications of weekly autocorrelations, which helped us quickly find the correct coefficients for fitting an ARIMA (Autoregressive Integrated Moving Average) model and decomposing the time series. These results are further described in the Results section.

It is worth noticing important dates. Next, a summary of important events is listed, taken from official announcements made available nationwide, but note that this list is not exhaustive and is listed here in chronological order.

- On February 27, 2020, Hugo López-Gatell Ramírez, head of the Undersecretaries of Prevention and Health Promotion at the Mexican Secretariat of Health, reported a patient in the INER (National Institute of Respiratory Diseases) as the first official COVID-19 case reported nationwide (https://twitter.com/HLGatell/status/1233245568668966913).
- On March 17, 2020, the number of cases had surpassed over 100, with 118 cases reported, marking an increment of 26% over the previous day. On this day, the first fatal COVID-19 case was also reported.
- On March 24, 2020, phase 2 of the pandemic evolution was officially started; that is, local transmission is observed between persons not in contact with foreigners. López-Gatell remarked that we are still observing transmissions, and the expectation is not to put an immediate end to the pandemic. I want to be clear that the success of a transmission reduction, instead of taking us to a shorter pandemic, will take us to a longer pandemic, but this is important in allowing for risk management. It means that each day, there are fewer cases than those that can be treated by the health system in Mexico.
- On April 21, 2020, phase 3 of the pandemic evolution starts, which maintains the safe-distance policies at least until May 30tĥ. This phase is also known as the epidemiological phase, which is characterized by having many cases in different localities, requiring strict health measurements, such as a general lockdown.
- On May 14, 2020, phase 1 of the recovery plan starts, lifting health restrictions in 269 municipalities where no official cases had been reported. Entrance to these municipalities is restricted.
- On May 15, 2020, the Mexican president addressed the nation concerning increased cases of domestic violence, which he flagged as up to 90% of such reports as false. Official reports do mark a large increase in domestic violence, averaging 11.2 deaths caused by domestic violence per day.
- On May 17, 2020, phase 2 of the recovery plan starts, allowing commercial activities for essential activities. The essential commercial activities are construction, mining, and automotive manufacturing. Each private company is responsible for designing, implementing, and operating the safety protocols they deem fit.
- On June 01, 2020, phase 3 of the recovery plan starts, allowing the opening of nonessential activities with all states in red status. A weekly *“traffic light”* system is implemented in each region, which depends on the health restrictions implemented and the reported cases. A red status allows for only essential activities to remain in operation.
- On June 23, 2020, a large earthquake was registered with an epicenter 23 Km south of Crucecita, Oaxaca. The United States Geological Service estimates that it had a magnitude of 7.4Mw.
- On July 15, 2020, it was reported that 800 public servants have passed away, of which only 273 were reported to be COVID-19 related.
- On August 13, 2020, over 500,000 cases were officially confirmed.
- On September 15, 2020, the Mexican president celebrates Independence day with no public. However, local celebrations depend on the local government, many of which did not follow this example.
- On October 05, 2020, the official methodology to record COVID-19 cases, and deaths, is updated in order to allow introducing old data into the records. This changes the official death count to 81,877 cases.
- On November 14, 2020, a total of 1,000,000 COVID-19 cases were officially confirmed.
- On November 20, 2020, a total of 100,000 COVID-19-related deaths were officially confirmed.
- On December 02, 2020, a contract was signed with private pharmaceutical Pfizer to acquire 34.4 million COVID-19 vaccines. It is expected to receive the first 250,000 vaccines this same month, which will be dedicated to health professionals.
- On December 11, 2020, the COFEPRIS (Federal Commission for Health Risks Protection) approved the emergency application of Pfizer's vaccines as long as they are utilized in accordance with the national vaccination policy.

We expect to find changes in the sentiments during these events, but keep in mind that it is possible there are other events not listed here, such as holidays or local festivities. The time series is shown in detail in the *Results* section.

## 4. Results

We performed sentiment analysis on COVID-19-related tweets posted in Mexico, from February 1, 2020, to December 31, 2020, forming a corpus of 760,064,879 tweets, which after preprocessing and filtering came to a total of *n*=2,142,890 utilized tweets retrieved from the *COVID-19 Twitter chatter dataset*. We performed a time series analysis to discover trends, seasonality, and other insights we might gain from the data, such as if there was an impact of changing policies on the emotional health of the Mexican population.

Figure 3 shows smoothed time series of the average sentiment polarity for the day and its variance. We can observe clear trends in the data, making clear that government policies do affect the general population mood. A clear example is the date when the WHO (World Health Organization) declared the COVID-19 a global pandemic, showing a negative peak in the mood trend immediately afterwards. Another example is when the government decided to put an early end to the lockdown in order to promote the local economy. After this decision, it is clear that there is controversy from the population, which can be observed by the increased variance in Figure 3, but in general showcasing increased peaks, both negative and positive. There are also clear negative peaks that correspond to either an official holiday or otherwise an economic-promoting activity, from which the official statement was that it was safe for the population to go out and gather in large numbers. This decision was received with heavy criticism from the general population, as is shown by the increased variance in Figure 3, resulting in a negative impact on the physical health, exposing a larger segment directly to the virus and thus increasing the infection and mortality rate.

Besides, Figure 3 highlights several relevant dates during the pandemic, using the labels [*a* … *q*], which are defined in the experiments section. Note that the list focuses on official national announcements only. Another point to note is the change in tweet volume. In February, that is, before the declaration of the pandemic, the average tweet volume in Mexico was 20,971 per day, adding to a total of 608,170 tweets for the month. March presented an average of 46,767 tweets per day and a total of 1,449,768 tweets for the month alone. This represents an increase in the volume of 238.382% between these two months.

The partial autocorrelation function, shown in Figure 4, indicates a strong correlation with the time series and makes an early estimation for the possible coefficients for fitting a statistical model. While the objective of this study is not to perform forecasting, but to describe the series, this early test indicates that there are valuable information to gain and an early indication of seasonality, for the correlation repeats itself weekly, as was also observed by [12]. This is confirmed by the Box–Pierce test, which yields a very small *p*-value (of 2.2*e*^−16^), suggesting a strong correlation.

The different components of the time series analysis, shown in Figure 5, show a slightly positive trend during the long-term lockdown. There is a slight and relatively constant slope during this period (*m*=0.0001110643).

Early indications of the partial autocorrelation function were found to be true, and there is a weekly seasonality, but it is curious to find no monthly or quarterly seasonality. Fitting a linear model to the trend shown leads to a negative intersection with a near-zero slope (*y*=−2.2087107971+0.0001110643*x*). However, Figure 3 shows a drastic change in the variance at the beginning of May, thus showing an increase in the controversy caused by the decrease of the mandatory lockdown followed by no clear guidelines on the part of the authorities.

## 5. Conclusion

We analyzed the sentiment polarity of COVID-19 related tweets gathered from February to December 2020 in Mexico. VADER was used as a sentiment analyzer, selected for its robustness and fast classification, and performed sentiment analysis on these data. To enable this, we have designed a flexible software architecture that, besides handling large datasets and dynamically adjusting scale, allows switching between language models and data sources in a timely manner. The technical solution utilizes microtriggers and serverless architecture to produce and process a data stream with the modularity of a single tweet, allowing easily changing the tweets' source to analyze other events and provide near real-time data. The same is true for the preprocessing and the language model utilized to calculate the tweet's sentiment polarity.

This study remarks on the impact of the pandemic and the decisions made by the national government and their official communications into the overall psychological well-being of the population. As such, it is important to highlight the essential need for a tool capable of providing feedback on time, considering the public's health, that is capable of drawing conclusions from large amounts of data in a short time. It is thus of great importance to incorporate this emotional well-being information as a feedback loop, and it to be adopted and utilized by decision-making organizations. This can greatly impact the decisions made by organizations of any size, showcasing in this study a national-wide impact of such decisions. And while emotional health is not the only metric that should be considered, this emotional feedback shows the public's perception and well-being, and it does provide a faster feedback loop than other regular pandemic-related metrics, which can take up to two weeks to manifest.

Nevertheless, this research opted for a somewhat different methodology to answer slightly different questions than those summarized in Table 2, which showcases other studies of COVID-19 related tweets. Among the key differences in this study is the study's span of a year-long worth of data, the use of the publicly available dataset, focusing the geographical area of study to that of Mexico, including tweets in both English and Spanish, a time series analysis to measure the evolution of the public perception of the pandemic, and striping down all the metadata available, making impossible analyzing individual's timelines by respecting user's privacy and keeping security as one of the guiding principles of the technical design.

There are some limitations in this study that are worth discussing. The study is restricted to a single country, Mexico. Still, the technology and methodology can be applied to a larger geographical region by simply feeding the system a more significant portion of the dataset or a different collection of tweets and using the same methodology this study performs. We utilized VADER as a language model for its versatility and well-studied behavior in other similar studies. However, different robust language models' architectures are worth exploring. The sentiment taxonomy utilized was the standard binary class classification, limiting the results to a single positive to negative dimension. While this produced interesting results, adopting a more robust language model would allow exploring a multiclass taxonomy. Another limitation is the striping of all metadata to ensure privacy and security while also preventing the making of a more extensive data analysis.

In the future, we want to focus on building publicly available dashboards that show the analysis results, and they could be used as a decision-making support tool. We have already developed tools that can scale out to different countries. However, this study utilized a corpus restricted to a single country, Mexico, and can easily modify these tools to adopt more complex sentiment taxonomies. We followed the standard practice of using a binary class sentiment classification taxonomy. Another area of interest would be comparing the results obtained in this study versus a more robust language model and exploiting the advantages of using modern machine learning architectures. However, this study can be utilized as a good baseline for performance in real-world tasks utilizing actual data. It is important to remark that we discarded all metadata included in the tweets, keeping users' privacy and security guiding design principles. This last point could enable more extensive, more sophisticated future studies, and to this end, the anonymous data are publicly available.

We have shown in this study the importance of having tools for visualizing sentiment polarity, which we performed on Mexican tweets related to COVID-19, which highlighted the impact of several policy decisions on the general's populations emotional health. This is essential, particularly during a health emergency such as this ongoing pandemic.

From February 1 to December 31, 2020, the overall sentiment polarity trend is constant and stable. Moreover, the sentiment polarity time series shows several events with a negative impact on the sentiment of the general population, showing a natural positive evolution until it stabilizes with an overall slope of 0.0001110643.

## Figures and Tables

**Figure 1:** *Data Consumption and Processing Overview.* The data are processed in three main stages: first, we load the desired Tweet IDs [6], then we consult them directly from Twitter using the official APIs. For preprocessing, we clean up and filter the data; then, we process this dataset in order to produce a time series of the perceived COVID-19-related sentiment. The data exploration and analysis are explained in detail sections *Sentiment Analysis of the Emotional Response to the COVID-19 Pandemic in Mexico* and *Procedure*.

**Figure 2:** *General Architecture Implemented in Google Cloud Platform (GCP).* This cloud-based architecture ingests tweets using the official Twitter APIs, sending each one of these through Google's Pub/Sub, which uses as endpoints basic preprocessing, raw storage, and a serverless function to calculate the sentiment polarity. The results of this function are fed into BigTable through another Pub/Sub pipeline.

**Figure 3:** COVID-19-related tweets average sentiment polarity per day in Mexico, including both the daily polarity average (top) and the daily variance (bottom), marking as well a few important dates, going with the labels [*a* … *q*]. The definition of each label, and its associated event, is described in the experiments section.

**Figure 4:** *Partial Autocorrelation Function (ACF) of the daily average of sentiment polarity of tweets.* This function is useful as an early indication of astrong autocorrelation present in the time series and provides estimations for the coefficients used in the time series analysis statistical model.

**Figure 5:** COVID-19-related tweets average sentiment polarity per day in Mexico. Here, we present the components of the time series analysis in the order shown: observations (mean polarity, similar to 3, trend in the time series, seasonality, and noise). We observe weekly seasonality, which is aligned with observed usage and mood patterns of Twitter by [12].

**Table 1:** Summary of massively distributed systems for performing sentiment analysis over large volumes of tweets.

Reference	Tech	Batch/stream	Features	Comments
Victor and Lijo, 2019 [13]	Hadoop & Spark	Both	HBase interface	
Sathya et al., 2019 [14]	Hadoop	Batch	Classifier selection, preprocessing, sarcasm, VR	Open source, needs self-hosting
Bhuvaneswari et al., 2019 [2]	Hadoop & Kafka	Both	Uses flume	
Cenni et al., 2018 [7]	Hadoop	Batch	—	Aggregation of 4 projects
Sehgal and Agarwal, 2016 [15]	Hadoop	Batch	—	
Kumar and Kala, 2016 [16]	Mahout	Batch	—	Less complex to build, experiments made on a single node
Kumamoto, Wada, and Suzuki, 2014 [17]		Batch	Graphs	No details
Khuc et al., 2012 [18]	Hadoop	Batch	HBase interface	Nice UI for data cleanup
Marcus et al., 2011 [19]	Hadoop	Batch	Peak detection, subevent selection	
*This study*	Microservices	Both	Autoscaling, easy to consume, cloud-native	Uses remote hosting

**Table 2:** Summary of similar studies following sentiment polarity over COVID-19 related tweets.

First author, ref	Summary	DataSet		
		Location	Time span (in 2020)	*n*
Adikari et al. [20]	Topic analysis follows popular subjects, pre/post lockdown	Australia	Jan to Sep	73K
Abd-Alrazaq et al. [21]	Uses PostgreSQL and topic analysis, pre/post lockdown		Feb 2 to Mar 15	167K
Boon-Itt and skunkan [22]	Topic analysis, 3 panel data analysis	US	Dec 13 to Mar 9	108K
Lwin et al. [23]	Uses the Plutchik basic sentiments, pre/post lockdown	Global	Jan 28 to Apr 9	20M
Xue et al. [24]	Topic analysis, pre/post lockdown	US	Mar 7 to Apr 21	4M
Valdez et al. [25]	Topic analysis, pre/post lockdown, follows popular subjects	US	Jan 28 to Apr 7	86M
Huerta et al. [26]	Pre/post lockdown	Ma, US	Jan 1 to May 14	2.88 M
*This study*	Time series, both Spanish and English	Mexico	Feb 1 to Dec 31	760M

**Table 3:** Monthly summary general sentiment polarity, between −1 and 1.

month	Mean	Median	Variance
February	−0.161653	−0.279797	0.166135
March	−0.180352	−0.296000	0.171638
April	−0.175834	−0.286133	0.186721
May	−0.135060	−0.266584	0.227397
June	−0.187039	−0.302487	0.214230
July	−0.171287	−0.296000	0.216006
August	−0.156576	−0.283995	0.220971
September	−0.137832	−0.284002	0.231412
October	−0.144219	−0.277552	0.223694
November	−0.157551	−0.283380	0.216210
December	−0.133056	−0.281765	0.228512

**Table 4:** Partial ACF (Autocorrelation Function) of the sentiment polarity time series.

Lag	Partial ACF
1	0.888493947
2	−0.188964510
3	−0.119674873
4	−0.030455558
5	−0.059030857
6	−0.009066172
7	−0.074336784
8	0.483162228
9	−0.174833350
10	−0.106022420
11	−0.042640744
12	0.036015376
13	−0.001715747
14	−0.022592658
15	0.262433976
16	−0.113870361
17	0.014280624
18	−0.095572696
19	0.040884337
20	−0.050324985
21	0.007294918
22	0.183424253
23	−0.077040062
24	−0.088658363
25	−0.023658966

## Data Availability

The data that support the findings of this study are available upon request to the corresponding author.
